# Big Data Recommendation Research Based on Travel Consumer Sentiment Analysis

**DOI:** 10.3389/fpsyg.2022.857292

**Published:** 2022-02-28

**Authors:** Zhu Yuan

**Affiliations:** School of Business, Jilin Business and Technology College, ChangChun, China

**Keywords:** tourism consumption, sentiment analysis, big data analysis, support vector machine, Map-Reduce

## Abstract

More and more tourists are sharing their travel feelings and posting their real experiences on the Internet, generating tourism big data. Online travel reviews can fully reflect tourists’ emotions, and mining and analyzing them can provide insight into the value of them. In order to analyze the potential value of online travel reviews by using big data technology and machine learning technology, this paper proposes an improved support vector machine (SVM) algorithm based on travel consumer sentiment analysis and builds an Hadoop Distributed File System (HDFS) system based on Map-Reduce model. Firstly, Internet travel reviews are pre-processed for sentiment analysis of the review text. Secondly, an improved SVM algorithm is proposed based on the main features of linear classification and kernel functions, so as to improve the accuracy of sentiment word classification. Then, HDFS data nodes are deployed on the basis of Hadoop platform with the actual tourism application context. And based on the Map-Reduce programming model, the map function and reduce function are designed and implemented, which greatly improves the possibility of parallel processing and reduces the time consumption at the same time. Finally, an improved SVM algorithm is implemented under the built Hadoop platform. The test results show that online travel reviews can be an important data source for travel big data recommendation, and the proposed method can quickly and accurately achieve travel sentiment classification.

## Introduction

In the era of big data, the whole tourism industry is also undergoing a revolution. As the scale of tourism development continues to grow, tourism data information is also exploding. Currently, big data are gaining more attention as it continues to integrate with the tourism industry, opening new doors for innovation in tourism decision making as well. Through mobile Internet technology, tourists can search for travel information, book travel services, and share travel experiences, generating “tourism big data.” In particular, in recent years, more and more travel consumers are making online travel reviews, which are comments on various aspects, such as services and prices (Boley et al., 2018; Buttazzoni et al., 2018; Cottrill et al., 2018; Luo et al., 2018; Prem et al., 2018; Yunlong and Yuanchang, 2018). The textual keywords are the most important data carriers of this information. By analyzing these textual reviews, it is possible to effectively understand the emotional state of consumers when traveling and their satisfaction with the service.

Online comment data are an important part of tourism big data, which have attracted extensive research because it can directly reflect the real emotions of tourists. The effects of tourism big data are mainly reflected in two aspects (Yi et al., 2014; Cynarski, 2018; Mayer and Woltering, 2018; Woosnam et al., 2018): on the one hand, tourism big data are beneficial to the transformation of tourism industry and have a great impact on the healthy and rapid development of tourism. On the other hand, tourism big data can contribute to the innovation of tourism management tools. “Sentiment analysis” takes textual comments as the object of research and is able to automatically determine the emotional tendencies of the subject of the comment. There are two main branches of sentiment analysis technology (De Vos, 2019; Haynes, 2020; Hunold et al., 2020; Van and Hieu, 2020), namely, sentiment analysis based on machine learning and sentiment analysis based on semantic methods. The former can rely on certain algorithms to achieve intelligent classification of data by computers. The main intelligent classification methods are Bayesian classification, KNN classification methods, decision tree classification, and support vector machine (SVM) classification. There are many other text classification algorithms, such as text classification using neural network approach. Abubakar and Ilkan (2016) pointed out that online reviews of tourist destinations affect tourists’ trust and stimulate their purchase demand. Gao et al. (2016) achieved affective polarity classification of text by building semantic features and binary models for sentiment analysis of microblog comment data. In addition, data mining and applications of sentiment analysis in tourism have been gradually developed. Tu and Tang (2016) pointed out the shortcomings of machine learning-based sentiment analysis methods in analyzing tourism reviews and established a sentiment analysis model based on semantic lexicon, which effectively improved the management efficiency of tourists’ evaluation remarks. Ma et al. (2016) constructed a sentiment analysis model, which is conducive to improving the service quality and image marketing of tourist destinations.

Although online review data have many advantages, its variable quantity and variety of characteristics also bring great trouble to the practical application. In particular, the current analysis and extraction technology are still immature, with low accuracy, slow extraction speed, and other drawbacks. Therefore, the current technology can no longer meet the needs of the market, so this problem needs to be solved. It should be noted that the current technology for processing online review data mainly relies on the concurrent storage and processing technology of massive data. HDFS concurrent storage system and Map-Reduce model have the ability to store and process massive data information at high speed concurrently (Fujiu et al., 2016; Rossini et al., 2016; Seera and Taruna, 2018; Sengan et al., 2020), which maximizes the use of all aspects of computer resources and has strong concurrency and high efficiency. SVM algorithm is a vector-based binary classification algorithm that is suitable for classification and analysis in massive data.

Therefore, this paper proposes an SVM classification solution based on the concurrent processing technology of massive data, and also designs and implements a classifier based on the improved SVM algorithm in the context of big data. The main work of this paper is reflected in the following two points: (1) This paper obtains standardized text data by word separation of travel reviews, so as to exploit the value of travel online reviews by using sentiment analysis technology, and makes an innovative exploration in the application. (2) The key technology for analysis of sentiment vocabulary is classification; therefore, this paper proposes to classify sentiment of travel online review data by machine learning algorithm and designs an improved SVM algorithm. The improved SVM algorithm makes full use of the threshold between SVM and point vector for denoising, which improves the accuracy of the system. Meanwhile, the Map-Reduce model in Hadoop platform is utilized to greatly improve the possibility of parallel processing and reduce the time consumption.

The rest of the paper is organized as follows: In section 2, the text pre-processing of online travel comment data is studied in detail, while section 3 provides the detailed classification model of tourism emotion based on machine learning. Section 4 provides detailed results and discussion. Finally, the paper is concluded in section 5.

## Text Pre-Processing of Travel Online Review Data

### Comment Type Information Pre-processing

The research data in this paper are mainly taken from the raw data of online travel platforms and microblogs. To convert these raw data into a language that can be recognized by computers, a systematic pre-processing work has to be performed. This specifically includes denoising, normalizing the representation, and word separation.

1. Denoising is to reduce data interference and make the study more focused. The objects removed by denoising are interfering comments and duplicate comments in the original comment data. Interference information is information that is not related to the research topic, such as “…” Such pure symbols do not reflect the commenter’s expression intention and have little value to the research topic, so this paper chooses to remove them. Repeated comments are multiple copies of the same comment by a certain user, so only one comment by this user is kept as the object of analysis in this paper.
2. The normative representation is mainly to correct and transform the original data so that it can be identified quickly in the data analysis. Since some commenters will adopt personalized expressions or Internet phrases in their comments, even the most common word separation system cannot identify them. Therefore, this paper will choose to replace or modify these data by consent to make the expressions more standardized and uniform.
3. The role of the word separation module is to make the evaluation dimensions correspond to the evaluation words one by one by using the word separation software, forming the initial correspondence-type data, and paving the way for the subsequent vectorization of the data.

Assuming that the vocabulary of the current evaluation dimension consists of *i* characters, match the first *i* characters of the current string. It also matches the *i* characters after the evaluation dimension (*i* values are 2–10). If this *i* character is the evaluation vocabulary, the field is sliced out and corresponds to the previous evaluation dimension, thus forming the initial correspondence data.

### Text Vectorization

When the corresponding data are formed, the vectorization process begins. The model can also be represented by the mathematical formula (Minaee et al., 2021):


(1) $$D=\left\{t_{1},w_{1};t_{2},w_{2};\ldots ;t_{n},w_{n}\right\}$$

where *D* is the set of feature terms, *t_n_* is each feature term, and *W_n_* is the weight corresponding to each feature term.

The specific process of data vectorization is divided into two parts: data vectorization and error tolerance (Hartmann et al., 2019).

#### Data Vectorization

The key to data vectorization is the determination of evaluation dimensions and evaluation vocabulary weights, and the frequency of dimension vocabulary occurrence is found to be a very scientific way of description through the preliminary market research, so the frequency value is chosen as the evaluation criterion here (Kadhim, 2019). The introduction of this evaluation dimension in the vector will play a crucial role in the classification results. When the vector is classified, based on the positive and negative values of the third component of the vector it will be possible to prioritize the comments into positive and negative, which will then be subdivided by the SVM algorithm, thus saving a lot of time costs and improving the efficiency of the system. For example, Table 1 shows the matching results of the travel-based sentiment evaluation. The effect after vectoring is shown in Table 2.

**Table 1:** Matching results of tourism-based emotional evaluation.

Evaluation dimension	Weights	Score evaluation	Tendency
Clogging	20%	84	negative
Traps	15%	85	negative
Dirty and disordered	15%	81	negative
Help	20%	80	positive
Beautiful Scenery	15%	68	positive
Friendliness	15%	45	positive

**Table 2:** Vector table.

Vector number	1	2
1	(11,84,7)	(13,80,6)
2	(22,85,9)	(12,45,4)
3	(17,81,7)	(13,44,9)
4	(4,45,−8)	(3,9,4)
5	(13,45,−10)	(14,32,−5)
6	(26,24,50)	(15,3,−6)

#### Error Tolerance

Since the combination of Chinese vocabulary is very different and the computer has limited ability to recognize Chinese text vocabulary, there will be various errors misleading the final result during the data pre-processing. Therefore, in the error-tolerant stage, when there is data in the vector that exceeds the boundary value, this vector is decisively excluded as an error vector to improve the accuracy of the system data.

## Machine Learning-Based Travel Sentiment Classification Model

The machine learning-based travel sentiment classification model contains the entire process from data collection to recommendation classification, as shown in Figure 1.

**Figure 1:** Support vector machine (SVM)-based travel sentiment classification model.

### SVM Algorithm Improvement

The core of the SVM algorithm is to find the support vector and the optimal hyperplane (Varatharajan et al., 2018; Zeng et al., 2018; Hu et al., 2020), so the key problem is to find the interval threshold between the vector corresponding to the data points and the support vector. Many linearly indistinguishable scenarios often occur in practice. Therefore, the selection of the kernel function is a key for the linearly indistinguishable problem. Since the data volume of travel online reviews is too large and the dimensionality is relatively low, the selection of polynomial type kernel function is particularly suitable.

For the case of linear indivisibility, the innovation of this paper is to improve the operation method by expanding the point vector in the SVM classifier into individual sub-vectors and then substituting them into the polynomial in turn. The original polynomial kernel function is as:


(2) $$K\left(x,x_{i}\right)={\left[\left(x\cdot x_{i}\right)+1\right]}^{d}$$

The SVM classifier decision function when linearly indistinguishable is as:


(3) $$\left.f\left(x\right)=\mathrm{sgn}{\left(\overset{n}{\underset{i=1}{\sum }}\alpha_{i}y_{i}\left(x_{i}\;\cdot \;x\right)+1\right)}^{d}+b\right)$$

where *x* is the vector to be classified, *x_i_* is the support vector, and *x* is an *n*-dimensional vector in the calculation of this formula.

It is obvious that the total time complexity is as:


(4) $$f\left(m,n,d\right)=m\left(n+d\right)$$

It can be seen that *n* inner product calculations are performed during the operation and the number of times is *d*.

Therefore, the computational effort of the improved SVM algorithm is not related to the number of support vectors but to the spatial dimensionality of the study context and the order of the kernel function in the polynomial. The use of the improved SVM algorithm is particularly effective for the case of this paper where the number of vectors is large and the dimensionality and order are small and low. When computing the vectors, there is no effect on the selection of the classification results and the calculation of the threshold value because the spreading vectors of the point vectors are discarded. Only the normal vectors need to be substituted into the computation to perform the classification, so that the efficiency of the algorithm is greatly improved. The penalty function in the linearly indistinguishable case is as:


(5) $$\min\frac{1}{2}∥W{∥}^{2}+C\overset{R}{\underset{i=1}{\sum }}\varepsilon_{i},s.t.,y_{i}\left(w^{T}x_{i}+b\right)\geq 1-\varepsilon_{i},\varepsilon_{i}\geq 0$$

where *C* is a free parameter, and based on practical experience, *C* is set to 2 in this study. *R* is the number of vectors.

Another important issue, the choice of the order *d*-value has a great impact on the accuracy and time complexity of the kernel function. Regarding the effect of different *d*-value choices on the recognition rate of the algorithm, it is illustrated here by the experimental results shown in Table 3.

**Table 3:** Experimental results with different *d* value.

Order *d*	Recognition rate	Number of support vectors
2	0.987	355
3	0.934	299
4	0.955	270
5	0.919	248
6	0.923	234
7	0.910	255
8	0.933	211

In this paper, the data dimension is 3 and the number of training samples is 3,776 data points. The polynomial type kernel function is used, and the parameter *C* is 2. From Table 3, we can see that the data recognition rate is highest when *d* = 2, so the *d* of the polynomial kernel function is 2 in this study.

### Big Data Processing Module

When deploying an HDFS storage structure on a Hadoop platform, a Master is used as the host, which is responsible for the NameNode and JobTracker. Each Slave usually has a DateNode for storing data information and its backups, and executes Map tasks and Reduce tasks in conjunction with a local TaskTraker according to the application requirements. The design idea of the Map-Reduce model is shown in Figure 2.

**Figure 2:** Map-Reduce model design ideas.

The Map-Reduce framework treats the input of an application as a set of <key,{list of value} > keys and the <key,{list of value} > keys input to the Map function are raw vector form data, where key represents the evaluation dimension weights and {list of value} corresponds to the “evaluation vocabulary” and “positive/negative meaning,” respectively. When <key,value> is derived from the Map, it comes to the Reduce class, and the Reduce task starts to process the healthy values scattered in many different nodes. The Reduce function saves the classification results of each data node into different classifiers and counts the number and percentage of nodes in each classifier.

## Experiment and Result Analysis

### Experimental Environment and Data Sources

The PC environment used for the test experiment is Intel I7 processor, 16G RAM, Windows 10 operating system, Eclipse, and Matlab. The cooperation with an online tourism platform in terms of big data was conducted and the online review data were captured using the big data cloud computing service platform owned by it. In 2019, the total tourism revenue of Hangzhou city was 219.741 billion yuan, an increase of 12.72% year-on-year. This study used this platform to capture online review data of Hangzhou West Lake Scenic Area in 2019. There are two main types of these data: (1) microblog data, such as Sina Weibo and Tencent Weibo; (2) OTA online review data, such as Ctrip.com, GoWhere.com, and Tongcheng.com. The collected raw data are pre-processed, among which the most important work is to manually classify these data, and the obtained division results yield the dataset shown in Table 4.

**Table 4:** Results of the manual division of the West Lake Scenic Area online comments.

	Number of comments with negative meaning	Number of comments with positive meaning	Total
Training set	20,670	18,033	38,703
Testing set	16,145	11,578	27,723
Total	36,815	29,611	66,426

### Evaluation Indicators

Travel sentiment classification can be summarized as a matter of binary classification. Those that contain negative evaluations are not recommended reviews and those that do not contain negative evaluations are recommended reviews. In general, there are two major dimensions for the evaluation criteria of classification models, one is the accuracy of classification, and the other is the efficiency of classification. In this paper, we will compare the travel sentiment classification models from these two perspectives. The evaluation metrics of classification accuracy use recall, correctness, and precision. Among them, correctness is an evaluation of the degree of classification of correct results in the classification results; precision is the percentage of each correct classification target in its category; and recall is a metric to evaluate the proportion of the category of recall targets. These evaluation metrics are calculated as follows:


(6) $$ACC=\frac{\mathrm{TP}+\mathrm{TN}}{\mathrm{TP}+\mathrm{FN}+\mathrm{FP}+\mathrm{TN}}$$

(7) $$P\left(pos\right)=\frac{\mathrm{TP}}{\mathrm{TP}+\mathrm{FP}}$$

(8) $$R\left(pos\right)=\frac{\mathrm{TP}}{\mathrm{TP}+\mathrm{FN}}$$

(9) $$P\left(neg\right)=\frac{\mathrm{TN}}{\mathrm{TN}+\mathrm{FN}}$$

(10) $$R\left(neg\right)=\frac{\mathrm{TN}}{\mathrm{FP}+\mathrm{TN}}$$

### Performance Analysis of the Improved SVM Algorithm

To verify the superiority of the improved SVM algorithm with respect to the original algorithm, two aspects of accuracy and time consumption are verified separately.

Figure 3 represents the comparison of the result accuracy of the original SVM and the improved SVM algorithm. It can be seen that the original SVM algorithm is higher at small data size. However, when the data volume grows to more than 600 G, the accuracy gap between the two algorithms gradually decreases. When the data volume grows to more than 1 T, the accuracy rate of the original SVM algorithm starts to decline, while the accuracy rate of the improved SVM algorithm remains around 80%. It can be inferred that the accuracy of the improved SVM algorithm has been well stabilized in the context of big data.

**Figure 3:** The accuracy comparison results of the original SVM and improved SVM algorithm.

Figure 4 shows the result accuracy of the improved SVM algorithm in the Hadoop system. It can be seen that after the introduction of Hadoop platform, the result accuracy of the algorithm has improved, especially when dealing with large data. From Figure 4, we can see that the accuracy rate is maintained at about 80%, which is basically in line with the actual application requirements. A comparison of the time consumption of the improved SVM algorithm and the original SVM algorithm is shown in Figure 5.

**Figure 4:** The accuracy of improvement algorithms results under the background of big data.

**Figure 5:** The time-consuming comparison of two algorithms.

From Figure 5, it is clear that when the amount of data is small, there is no significant advantage of the improved SVM algorithm after decomposing the vectors due to the limited number of both point vectors and support vectors. Therefore, there will not be much difference between the two in terms of time cost. However, when the data size gradually increases, the improved SVM algorithm has a great advantage in the computation of kernel function due to the linear indistinguishability gradually increases, especially when the data size is more than 20 GB, this advantage is especially obvious. Overall, in the context of massive data, the improved SVM algorithm greatly improves the execution efficiency of the algorithm while ensuring a certain accuracy of the results.

### Performance Comparison of Different Classification Models

Sentiment analysis models based on SVM, plain Bayes and dictionary rules were continuously trained and optimized according to five major measures for assessing model accuracy. The classification results of different models at the same test set are shown in Table 5.

**Table 5:** Classification effects of different models at the same test set.

Algorithm	Number of test sets	*Acc*	*P*(*po*s)	*R*(*po*s)	*P*(*neg*)	*R*(*neg*)
Improved SVM	1,000	0.838	0.825	0.912	0.816	0.738
	5,000	0.874	0.883	0.919	0.859	0.803
	10,000	0.880	0.889	0.909	0.866	0.837
	15,000	0.880	0.875	0.907	0.886	0.847
	20,000	0.874	0.861	0.915	0.891	0.825
	27,723	0.870	0.856	0.915	0.890	0.817
NaiveBayes	1,000	0.838	0.836	0.895	0.842	0.762
	5,000	0.859	0.874	0.902	0.833	0.789
	10,000	0.866	0.878	0.898	0.849	0.821
	15,000	0.850	0.851	0.875	0.847	0.820
	20,000	0.846	0.844	0.878	0.848	0.807
	27,723	0.853	0.850	0.890	0.857	0.813
Dictionary	1,000	0.880	0.960	0.828	0.800	0.952
	5,000	0.845	0.900	0.811	0.790	0.888
	10,000	0.880	0.924	0.872	0.823	0.892
	15,000	0.855	0.930	0.836	0.753	0.889
	20,000	0.856	0.928	0.811	0.784	0.916
	27,723	0.867	0.931	0.841	0.790	0.906

The results of the accuracy analysis of these three models are shown in Figure 6. From the results, it can be seen that the commonality of the three is that the accuracy rate is high, above 83%, and all of them can achieve the accurate management of tourism emotion. However, there are still some differences among the three. Compared with the model based on sentiment dictionary rules, the classification accuracy of the machine learning-based model is more stable, and the improved SVM classifier is generally better than the plain Bayesian classifier. Among them, the classification accuracy of the dictionary model is higher than that of the machine learning classification when the number of test sets is small, but it gradually decreases as the number of test sets increases.

**Figure 6:** Sentiment classification accuracy (*Acc*) of each classifier.

In summary, the travel sentiment classification model based on sentiment dictionary has better classification results when dealing with a small amount of text. However, as the number of test sets increases, the improved support vector machine-based travel sentiment classification model is able to achieve more desirable classification results. Therefore, the improved support vector machine-based sentiment analysis method has great superiority in dealing with large amount of travel review data.

## Conclusion

In this paper, a typical method of sentiment analysis is used to build a machine learning model based on support vector machines to analyze the sentiment of travel online comments, and the feasibility and effectiveness of the idea are verified by experimental models. In the algorithm study, the SVM support vector machine algorithm is chosen and improved for the case of clear categories and large amount of data. In addition, the improved SVM algorithm is applied using Map-Reduce and classifies large-scale textual keywords, while the HDFS system is used to store and read and write data rows concurrently to improve the efficiency when training large amounts of data. Finally, the efficiency of the proposed method is verified through comparative experiments. The shortcoming of this study is that the data size of the test set used in the experiments is limited and does not reflect well the speedup ratio relationship of the classification process under more processors. The data size of the experiments and the number of nodes in the experimental platform will be increased in the future.

## Data Availability Statement

The raw data supporting the conclusions of this article will be made available by the authors, without undue reservation.

## Author Contributions

ZY was responsible for designing the framework of the entire manuscript from topic selection to solution to experimental verification.

## Conflict of Interest

The author declares that the research was conducted in the absence of any commercial or financial relationships that could be construed as a potential conflict of interest.

## Publisher’s Note

All claims expressed in this article are solely those of the authors and do not necessarily represent those of their affiliated organizations, or those of the publisher, the editors and the reviewers. Any product that may be evaluated in this article, or claim that may be made by its manufacturer, is not guaranteed or endorsed by the publisher.
